# Evaluation of the Health Situation among Recovered Cases of COVID-19 in West Bank, Palestine, and Their Onset/Recovery Time

**DOI:** 10.1155/2022/3431014

**Published:** 2022-03-21

**Authors:** Hani Naseef, Abdallah Damin Abukhalil, Tala Orabi, Mohammad Joza, Carmen Mashaala, Malak Elsheik, Aseel Dababat, Maram Qattosa, Ni'Meh Al-Shami

**Affiliations:** Department of Pharmacy, Nursing and Health Professions, Birzeit University, West Bank, State of Palestine

## Abstract

**Background and Aims:**

COVID-19 emerged at the end of 2019 and was classified as a global pandemic in March 2020. Infected cases of SARS-CoV-2 experience symptoms during initial infection 2–14 days after virus exposure, and some symptoms and complications may persist after recovery. This study evaluated the onset/recovery time, postrecovery symptoms, complications, and factors affecting the health situation of recovered cases of COVID-19 in West Bank, Palestine.

**Methods:**

This cross-sectional study was conducted using a questionnaire based on related scientific articles and expert recommendations. It was distributed to recovered COVID-19 patients either face-to-face or online. Chi-square and Fisher's exact tests were used to investigate the significant relationships. The data were analyzed using SPSS version 22. *Findings*. A total of 686 participants completed the questionnaire; the mean age was 28·1 ± 11·8. SARS-CoV-2 infection recovery time was 1–2 weeks in most participants. A total of 72·4% developed post-COVID-19 symptoms. Fatigue (260, 38.0%), loss of smell (224, 32.7%), headache (207, 30.7%), and joint pain (188, 27.4%) were the most reported postrecovery symptoms. In women, fatigue and headaches were the most common symptoms that persisted after recovery. Diabetic patients endured continuous muscle and joint pain. *Interpretation.* Patient health situation, recovery time, and symptoms post-COVID-19 infections are affected by many demographic factors and disease status.

## 1. Introduction

Coronavirus is a human virus that causes respiratory infections diseases such as SARS-CoV-2, known as COVID-19. COVID-19 has mainly caused respiratory infections that started in December 2019 in Wuhan, China, and has rapidly spread worldwide. Approximately 156 million cases were diagnosed, and approximately 134 million recovered by May 15, 2021 [1]. COVID-19 symptoms vary among individuals and range from mild to moderate to severe. Fatigue, dry cough, tiredness, loss of smell and taste, and headache are common symptoms. Furthermore, breathing difficulties, loss of speech and movement, and chest pain are considered serious ones [2–4]. The severe symptoms were found in patients over 60 years of age or those with concomitant diseases, such as hypertension, diabetes, heart, and respiratory problems. At the same time, mild-to-moderate symptoms were found in children and patients under 19 years [5].

The onset of an infection is the initial appearance of the disease signs and symptoms [6]. The median time from disease onset to recovery is 3–6 weeks for severe cases and 2 weeks for mild cases [7]. Although many people have recovered from the virus, many of them do not return to their everyday life; in other words, COVID-19 affects people's health in the long run, including heart muscle, heart failure, damaged lungs, mental problems, musculoskeletal problems, brain and nervous system damage, and blood vessel problems [8]. Some symptoms persist after recovery, such as fatigue, shortness of breath, loss of taste and smell, cough, and headaches [8].

A study conducted on 179 participants in Italy reported the persistence of at least one symptom in recovered patients with COVID-19. A total of 53·1% of subjects still experienced fatigue; 43·4% had continued dyspnea; 27·3% joint pain; and 21·7% experienced chest pain [8]. Another study conducted in Tours, France, revealed that 68% of participants had at least one symptom 30 days after symptoms onset; moreover, 66% of the patients were still suffering from the disease's symptoms, mainly ageusia anosmia, 60 days later. The same study showed that on day 30, 36·7% of patients were suffering from shortness of breath (dyspnea), and on day 60, 30% of patients reported dyspnea. In addition, 50% and 40% of patients reported fatigue and tiredness on days 30 and 60, respectively. The study also showed that participants who experienced symptoms at day 60 were hospitalized or had a severe COVID-19 infection [7]. Another study conducted by Columbia University hospital in May 2020 reported many persistent symptoms after COVID-19, such as fatigue, body aches, shortness of breath, headache, psychological problems such as depression, change in smell or taste, cough, and others [9]. A regional study in Egypt showed that fatigue was the most common symptom reported by participants post-COVID-19 infection [10]. In a systemic review of 69 studies on COVID-19 complications, Al-Jumaili et al. reported that many patients experienced lung abnormalities, exercise intolerance, and neurological problems [11]. By May 2021, about 300,000 cases were diagnosed in Palestine, and 281,000 recovered [1]. No studies have been conducted in Palestine to assess patients' health status post-COVID-19 infection. This study aimed to evaluate the onset/recovery time, postrecovery symptoms, complications, and factors affecting the health situation of recovered cases of COVID-19 in West Bank, Palestine.

## 2. Materials and Methods

### 2.1. Study Design and Sample

A questionnaire-based cross-sectional descriptive observational study was conducted from 21 December 2020 to 12 February 2021 in Palestine. The study included participants aged 18 years and older who were previously diagnosed with COVID-19 infection and recovered. The questionnaire was offered online or through in-person interviews.

The questionnaire was designed and provided by Google Forms (Google Inc., USA) under the supervision of the IT department personnel. The representative sample size of 382 was calculated based on the total recovered patients of COVID-19 from the West Bank with a 95% confidence level and a 5% accepted margin of error. The sample size was calculated by the Raosoft sample size calculator website using 63,881 cases (the total number of cases that were diagnosed in Palestine on 29 November 2020). In reference [12], 740 recovered cases participated. Fifty-four participants were excluded due to duplication, incomplete responses, or age under 18 years.

The IRB committee approved the study at the Faculty of Pharmacy, Nursing, and Health Professions, Birzeit University (reference number BZU-PNH-2006).

### 2.2. Study Tool

The questionnaire was developed based on a review of related research that represents a variety of post-COVID-19 symptoms, their duration, and its correlation with chronic diseases, age, gender, body mass index (BMI) [13], smoking status [14, 15], and blood groups [16, 17].

The researchers reviewed and evaluated the questionnaire components at different meetings. The questionnaire was reviewed by five multidisciplinary experts from the Faculty of Pharmacy, Nursing, and Health Professions. The questionnaire was modified accordingly based on the feedback received. Furthermore, it was translated into Arabic by experts.

A pilot study was conducted to ensure study validity and questionnaire consistency among 22 COVID-19 recovered patients. Participants were requested to complete the questionnaire and provide their feedback regarding its clarity, construction, and relevance. Based on the participants' assessments, some adjustments were made to the final Arabic draft.

The questionnaire included four sections related to the patients' health situation: demographics, quarantine, postrecovery symptoms, and symptom duration. These sections contained 23 questions formulated as open- and closed-ended multiple-choice questions. The demographic information section included 15 questions concerning age, gender, weight, height, place of residence, blood group, health, infectious, smoking, and pregnancy status. The quarantine section included 3 questions on place and duration. Finally, the postrecovery symptoms and duration section consisted of 5 questions addressing the type of symptoms during infection, postrecovery symptoms, their duration, and any associated physiological changes.

### 2.3. Statistical Analysis

All questions were coded and imported into IBM SPSS Statistics 22 for analysis. Descriptive statistics were used to analyze the data. First, questions were recorded and categorized; height and weight were computed to BMI and then categorized based on BMI classification: underweight (below 18.5), normal or healthy weight (18.5–24.9), overweight (25.0–29.9), and obese (≥30.0) [18]. Blood groups were categorized as unaccompanied by the Rhesus (Rh) factor (A, B, AB, and O). Next, categorization of symptom numbers for every participant was done, obtaining 0 symptoms, 1–8 symptoms, and 9–15 symptoms. Next, age was divided into five classes (18–20, 21–30, 31–40, 41–50, and ≥50). Finally, governorates were categorized as northwest, southwest, midwest, and Jerusalem.

Chi-square or Fisher's exact tests with a 95% confidence interval were performed to investigate the correlations between the demographics and symptoms and their duration.

## 3. Results

### 3.1. Demographic Information

A total of 740 participants completed the questionnaire; 690 completed the electronic Google Forms; and 50 completed the written survey. Unfortunately, 54 participants were excluded from the study because of incomplete surveys. Three hundred (43·7%) participants were between 21 and 30 years with a mean age of 28.1 ± 11.8. About two-thirds of the patients were females, 469 (68.4%). Tobacco smokers were 114 (16.6%), and 101 (14.7%) had chronic diseases. Furthermore, 26 (3.9%) were underweight; 362 (54.4%) were normal; 178 (26.8%) were overweight; and 99 (14.9%) were obese according to the body mass index (BMI). The percentages of participants who recovered from COVID-19 in 1–2 weeks were 482 (70.3%), and 133 (19.4%) took more than 2 weeks to recover. The most common blood type among the participants was blood group A, 28 (49.7%).  Table 1 presents the demographic backgrounds of the respondents who completed the survey.

### 3.2. Symptoms after Recovery and Their Duration

At least one post-COVID-19 symptoms continued to appear in 497 (72.4%) of the participants; 87 (12.7%) of the cases have had physiological changes after recovery. Fatigue, loss of smell, and headache were the most common symptoms that lasted after recovery, with percentages of 260 (38.0%), 224 (32.7%), and 207 (30.2%), respectively. The four main symptoms that lasted for more than one month were loss of smell, fatigue, headache, and joint pain, with a percentage of 74 (11.0%), 49 (7.2%), 36 (5.3%), and 43 (6.4%), respectively. Few patients, 87 (12.7%), reported physiological changes after recovery, such as parosmia, gastrointestinal changes, menstrual irregularities, rash, and coagulation changes (Table 2).

Table 3 shows chi-square test results for participant characteristics in relation to COVID-19 infection postrecovery symptoms. Female (364, 77.6%) were significantly (*p* < 0.001) more likely to complain from symptoms after recovery compared to males (133, 61.3%). No significant difference was found with the other characteristics: age, BMI, blood group, being a smoker, or suffering from chronic disease.

Fatigue, loss of smell, and headache were the main symptoms that lasted after recovery, with the prevalence for females 211 (42.9%), 163 (34.8%), and 162 (34.5%), respectively, and for males 59 (27.2%), 61 (28.1%), and 45 (20.7%), respectively. The *p*-value for gender was <0.0001 for fatigue and headache and 0.084 for loss of smell. As shown in Table 4, most participants, regardless of their age group, experienced symptoms after recovery. However, regarding the blood type, it is noticeable that participants with blood type B experienced the lowest symptoms after recovery was 46 (63.0%; Table 3). In addition, they showed the lowest percentages of fatigue, loss of smell, and headache after recovery, with 20 (27.4%), 24 (32.9%), and 14 (19.2%), respectively, compared to participants with other blood types.

### 3.3. Chronic Diseases and Symptoms after Recovery

As shown in Table 5, 74 (73.3%) of chronic disease cases had at least one symptom that continued after recovery (*p* value 0.842 (not significant)).

Muscle and joint pain were the most common significant symptoms among one-third of patients with chronic disease with a *p*-value of 0.0010, as shown in Table 6. Also, Table 7 shows that more than 70% of patients with hypertension, diabetes, high cholesterol, and heart disease suffered from at least one post-COVID-19 symptom.

Table 7 shows the prevalence of postrecovery symptoms among participants with chronic diseases. For example, 14 (34.1%) of participants with hypertension reported continued cough postrecovery with a *p*-value of 0.0070, and 10 (40.0%) of participants with diabetes experienced a loss of taste with a *p*-value of 0.036. On the other hand, 6 (42.9%) of patients with heart disease and atherosclerosis endured continued chest pain after recovery with a *p*-value of 0.0090, and 9 (56.3%) of high cholesterol cases experienced a loss of taste after testing negative for COVID-19 with a *p*-value of 0.0030.

## 4. Discussion

Emerging evidence has shown that many patients continue to suffer from complications or symptoms after SARS-CoV-2 infection recovery. In addition, patient characteristics such as gender, blood type, BMI, smoking history, and history of chronic disease might affect the patient's health during or after infection. According to the current study's data, 72·4% of the participants experienced at least one symptom after recovery. These findings align with those of previous studies in which many recovered patients experienced post-COVID-19 symptoms [10]. In addition, several studies have shown that most COVID-19 patients have suffered from long COVID-19 such as fatigue, headache, loss of smell and taste, cough, and body aches [7–9, 11, 19].

In this study, postrecovery symptoms were more prevalent among females, with a percentage of 77.6% versus 61.3% in males. This finding is supported by other studies in which females continued to experience symptoms postrecovery [20–22]. However, other participant characteristics, such as age, BMI, smoking status, and blood groups, showed no correlation with postrecovery symptoms. This finding contraindicates other studies where A and AB blood types have a higher risk of experiencing severe COVID-19 symptoms [16, 23], and higher BMI increases the risk of severe COVID-19 [24]. Also, studies have shown that elderly patients experience more severe symptoms during infection [25].

Fatigue, loss of smell, and headaches were the most common symptoms after recovery. Different studies confirmed fatigue and headache [8, 10]. In addition, the results revealed that females had had these symptoms more frequently. These results align with different studies in which females were more associated with fatigue after recovery than males [26]. Females experienced more loss of smell symptoms than males during infection [27]. A study in the USA showed that headache was more prevalent in females during infection [28]. Furthermore, age was statistically significant with persistent fatigue, indicating fatigue persisted more frequently in elderly patients and more affected by COVID-19 symptoms [25].

Patients with chronic disease and COVID-19 infection continue to be challenging for healthcare providers, as information about the effects of the virus on body systems is still evolving. Surprisingly, this study showed that chronic diseases did not affect the continuity of COVID-19 symptoms, even though various studies have shown that chronic diseases increase infection risk, mortality, and severity [29, 30]. The most common significant symptoms associated with various chronic diseases are muscle and joint pain.

Certain post-COVID-19 symptoms were associated with specific chronic diseases, such as hypertension patients experienced persistent cough, diabetes patients experienced continued loss of taste; this might be because diabetes mellitus causes taste disturbances, and COVID-19 could worsen [31]. Heart disease and atherosclerosis have been linked to post-COVID-19 chest pain, which could be due to the complications of these diseases [32]. However, high cholesterol patients reported a loss of taste after recovery related to uncontrolled or high serum cholesterol, which has been associated with taste disorder [33], and COVID-19 might aggravate this symptom and make recovery more complex.

More than two-thirds of the subjects needed one to two weeks to recover from the virus (to have a negative COVID-19 test), according to multiple studies, and the virus takes one to two weeks to exist in the body for moderate instances and six weeks for severe cases [34, 35].

## 5. Conclusion

In this study, the recovery time among the participants was between one and two weeks. Fatigue, headache, and loss of smell are the most common symptoms reported post-COVID-19 infection. Symptom duration was longer in females. In addition, fatigue is the most common symptom reported in elderly patients post-COVID-19. Finally, various chronic diseases contribute to specific persistent symptoms after recovery, such as hypertension patients experiencing persistent cough, diabetes, and high cholesterol patients experiencing persistent loss of taste, and heart disease and atherosclerosis patients experiencing persistent chest pain. COVID-19 infection, symptoms, complications, duration, treatment, and vaccination continue to be the twenty-first-century health and science puzzle requiring much effort and research from the scientific community to uncover this disease and end the pandemic.

## 6. Limitations

This study had several limitations. There was insufficient data for specific groups, such as old age and chronic disease patients. In addition, some patients who completed the questionnaire might have had recall bias and the use of convenience sampling.

## Figures and Tables

**Table 1:** Demographic information.

Variable	Categorization		Count (frequencies)		Percentage (%)
Age	18–20		193		28.1
	21–30		300		43.7
	31–40		62		9
	41–49		72		10.5
	>50		59		8.6
Sex	Male		217		31.6
	Female		469		68.4
Smoking (cigarettes and shisha)	Nonsmoker		572		83.4
	Smoker		114		16.6
Pregnancy (females)	Yes		10		1.5
	No		467		68.1
Chronic diseases	Yes		101		14.7
	No		585		85.3
Hypertension	Yes		41		6
	No		625		94
Diabetes	Yes		25		3.6
	No		661		96.4
Heart diseases and atherosclerosis	Yes		14		2
	No		672		98
Cholesterol	Yes		16		2.3
	No		669		97.7
Obesity	Yes		99		14.4
	No		587		85.6
BMI categorization	UWT^a^		26		3.9
	Normal weight		362		54.4
	OWT^b^		178		26.8
	Obese		99		14.9
Governorates	NWB^c^		163		23.8
	MWB^d^		278		40.5
	SWB^e^		104		15.2
	Jerusalem		141		20.6
Blood categorization	A		280		49.7
	B		73		13.0
	AB		52		9.2
	O		158		28.1
How long have you had coronavirus?	Less than a week		71		10.3
	One to two weeks		482		70.3
	More than two weeks		133		19.4
How long has it been since you recovered from COVID-19?	Less than a week		197		28.7
	From a week to a month		246		35.9
	From a month to three months		144		21.0
	From three months to six months		92		13.4
	More than six months		7		1
Were you in quarantine^f^?		Yes		652	95
		No		34	5

*Note.* ^a^Underweight, ^b^overweight, ^c^north West Bank, ^d^middle West Bank, ^e^south West Bank, and ^f^a place where infected people get isolated.

**Table 2:** Symptoms after recovery.

Variable	Categorization	Frequency	Percentage (%)
Physiological change after recovery	Yes	87	12.7
	No	599	87.3
Symptoms after infection	Yes	497	72.4
	No	189	27.6
Symptoms persisted after recovery			
Fatigue		260	38.0
Loss of smell		224	32.7
Headache		207	30.2
Joint pain		188	27.4
Back pain		169	24.6
Muscle pain		159	23.2
Loss of taste		156	22.7
Lack of focus		147	21.5
Cough		126	18.4
Anxiety and tension		118	17.2
Chest pain		116	16.9
Shortness of breath		109	15.9
Eye pain		87	12.7
Loss of appetite		67	9.8

**Table 3:** Experiencing symptoms after recovery.

		Experienced symptoms after recovery	*p* value
Gender	Female	364 (77.6)	<0.0001
	Male	133 (61.3)	
Age (years)	**18–20**	133 (68.9)	0.27
	**21–30**	220 (73.3)	
	**31–40**	45 (72.6)	
	**41–50**	59 (81.9)	
	>50	40 (67.8)	
Chronic disease	Yes	74 (73.3)	0.84
	No	423 (72.3)	
Blood categorization	A	209 (74.6)	0.71
	B	46 (63.0)	
	AB	43 (82.7)	
	O	120 (75.9)	
Smoker	Yes	78 (68.4)	0.29
	No	419 (73.3)	
BMI	Underweight	18 (69.2)	0.23
	Normal	265 (73.2)	
	Overweight	120 (67.4)	
	Obese	78 (78.8)	

*Note.* Chi-square test was used; the significant value is less than 0.05.

**Table 4:** The common symptoms after recovery.

Variable		Fatigue, *n* (%)	*p*-value	Loss of smell, *n* (%)	*p* value	Headache, *n* (%)	*p* value
Gender	Female	211 (42.9)	<0.0001	163 (34.8)	0.084	162 (34.5)	<0.0001
	Male	59 (27.2)		61 (28.1)		45 (20.7)	
Age (years)	18–20	59 (30.6)	0.0050	61 (31.6)	0.38	58 (30.1)	0.83
	21–30	108 (36.1)		107 (35.4)		95 (31.7)	
	31–40	31 (50.0)		21 (33.9)		16 (25.8)	
	41–50	37 (51.4)		22 (30.6)		19 (26.4)	
	>50	25 (42.4)		13 (22.0)		19 (32.2)	
Diabetes	Yes	10 (40.0)	0.83	12 (48.0)	0.096	8 (32.0)	0.84
	No	250 (37.9)		212 (32.1)		199 (30.1)	
Hypertension	Yes	19 (46.3)	0.25	13 (31.7)	0.89	16 (39.0)	0.20
	No	241 (37.4)		207 (32.7)		191 (29.6)	
Cholesterol	Yes	7 (43.8)	0.63	8 (50.0)	0.13	5 (31.3)	1.00
	No	253 (37.9)		215 (32.1)		201 (30.0)	
Heart diseases and atherosclerosis	Yes	5 (35.7)	0.86	3 (21.4)	0.57	5 (35.7)	0.77
	No	255 (38.0)		221 (32.9)		202 (30.1)	
Blood categorization	A	113 (40.4)	0.12	94 (33.6)	0.95	84 (30.4)	0.070
	B	20 (27.4)		24 (32.9)		14 (19.2)	
	AB	24 (46.2)		19 (36.5)		18 (34.6)	
	O	66 (41.8)		56 (35.4)		57 (36.1)	
Smoker	Yes	38 (33.3)	0.27	43 (37.7)	0.21	28 (24.6)	0.15
	No	222 (38.9)		181 (31.6)		179 (31.3)	
BMI	Underweight	10 (38.5)	0.22	11 (42.3)	0.43	11 (42.3)	0.33
	Normal	127 (35.2)		125 (34.5)		111 (30.7)	
	Overweight	64 (36.0)		53 (29.8)		46 (25.8)	
	Obese	46 (46.5)		29 (29.3)		29 (29.3)	

*Note.* Chi-square test was used; the significant value is less than 0.05.

**Table 5:** Chronic diseases and continuity of symptoms after recovery.

	Experienced symptoms		*p* value
Variable	Experienced symptom after recovery? *n* (%)		
Chronic disease	Yes	74 (73.3)	0.84
	No	423 (72.3)	

Variable	Experienced muscle pain after recovery? *n* (%)		
Chronic disease	Yes	36 (36.0)	0.0010
	No	123 (21.0)	

Variable	Experienced joint pain after recovery? *n* (%)		
Chronic disease	Yes	36 (35.6)	0.044
	No	152 (26.0)	

**Table 6:** Chronic diseases and the continuity of at least one post-COVID-19 symptom.

Disease	Frequency (%)
Hypertension	33 (80.5)
Diabetes	19 (76.0)
Cholesterol	13 (81.3)
Heart diseases and atherosclerosis	10 (71.4)

**Table 7:** Association of cardiovascular diseases, diabetes, and post-COVID-19 symptoms.

Chronic diseases and symptoms	Frequency (%)
Blood pressure and continued fatigue after recovery	19 (46.3)
Blood pressure and continued cough after recovery	14 (34.1) *p*-value **0.007**
Blood pressure and continued headache after recovery	16 (39.0)
Blood pressure and continued joint pain after recovery	16 (39.0)
Blood pressure and continued muscle pain after recovery	18 (43.9)
Blood pressure and continued back pain after recovery	14 (34.1)
Blood pressure and continued loss of smell after recovery	13 (31.7)
Diabetes and continued loss of taste after recovery	10 (40) *p*-value **0.036**
Diabetes and continued loss of smell after recovery	12 (48)
Diabetes and continued fatigue after recovery	10 (40)
Diabetes and continued joint pain after recovery	8 (32)
Heart diseases and atherosclerosis and continued fatigue after recovery	5 (35.7)
Heart diseases and atherosclerosis and continued headache after recovery	5 (35.7)
Heart diseases and atherosclerosis and continued lack of focus after recovery	5 (35.7)
Heart diseases and atherosclerosis and continued joint pain after recovery	5 (35.7)
Heart diseases and atherosclerosis and continued chest pain after recovery	6 (42.9) *p*-value **0.009**
Heart diseases and atherosclerosis and continued back pain after recovery	5 (35.7)
Cholesterol and continued cough after recovery	5 (31.3)
Cholesterol and continued loss of smell after recovery	8 (50.0)
Cholesterol and continued loss of taste after recovery	9 (56.3) *p*-value **0.003**
Cholesterol and continued fatigue after recovery	7 (43.8)
Cholesterol and continued shortness of breath after recovery	5 (31.3)
Cholesterol and continued headache after recovery	5 (31.3)
Cholesterol and continued joint pain after recovery	5 (31.3)
Cholesterol and continued muscle pain after recovery	6 (37.5)
Cholesterol and continued back pain after recovery	6 (37.5)

*Note.* Chi-square test was used; the significant value is less than 0.05.

**Table 8:** Demographic information.

D1	Age	
**D2**	Sex	1. Male and 2. Female
**D3**	Governorate	1. Ramallah and Al Bireh, 2. Jerusalem, 3. Bethlehem 2, 4. Tubas and Jenin, 5. Tulkarm, 6. Nablus, 7. Herbon, 8. Qalqilyah, 9. Salfit, and 10. Jericho
**D4**	Length	
**D5**	Weight	
**D6**	Blood type	1. A+, 2. A–, 3. B+, 4. B–, 5. AB+, 6. AB–, 7. O+, 8. O–, and 9. I do not know my blood type
**D7**	Do you have any chronic diseases?	1. No, 2. blood pressure, 3. diabetes, 4. heart diseases and/or atherosclerosis, 5. high cholesterol, 6. obesity, 7. cancer, and 8. other than that
**D8**	How long have you had coronavirus? (The period by which the test result was positive)	1. Less than a week 2. One to two weeks 3. More than two weeks
**D9**	How long has it been since you recovered from coronavirus? (After the appearance of a negative result of the PCR test for coronavirus or 14 days after the date of onset for corona infection)	1. Less than a week 2. Week to month 3. One to three months 4. Three to six months 5. More than six months
D10	Have you experienced any symptoms in general during your infection?	1. Yes 2. No
D11a	Are you a smoker?	1. Yes 2. No
D11b	If yes, how many cigarettes do you smoke every day?	
D11c	If yes, how long have you been smoking (in years)?	
D12a	Were you pregnant during the period of your infection?	1. Yes 2. No 3. Does not apply (male)
D12b	If yes, have you experienced premature labor?	1. Yes 2. No

*Note.* Recovery from coronavirus in this questionnaire is intended to show a negative result when performing a PCR test.

**Table 9:** Post-recovery symptoms and symptoms duration.

(S4) If the symptom is eliminated, how long did it take to get rid of it? Answer 1. Less than a week 2. Two to four weeks 3. More than a month	(S3) Describe the symptom intensity after recovery Answer 1. Light 2. Moderate 3. Severe	(S2) Did the symptom continue to appear even after recovering from the coronavirus? Answer: 1. Yes 2. No	(S1) Describe the symptom intensity during the infection Answer: 1. Light 2. Moderate 3. Severe	Symptoms
				(A) Fatigue
				(B) Cough
				(C) Loss of smell
				(D) Loss of taste
				(E) Shortness of breath
				(F) Headache
				(G) Loss of appetite
				(H) Fever
				(I) Anxiety and tension
				(J) Lack of focus
				(K) Joint pain
				(L) Muscle pain
				(M) Chest pain
				(N) Eyes pain
				(O) Back pain
1. Yes 2. No	Have you experienced any change in body function or an emergence of a new symptom after recovery from the virus?			S5A
	If yes, please specify the change that has occurred.			S5B

*Note*. (1) If any of these symptoms did not appear, please leave the answer boxes for this symptom blank. (2) When you reach the box (temperature): If your temperature was less than 37.5°C, leave the answer box blank. If your temperature was between 37.5 and 38°C, the intensity of this symptom is moderate. If your temperature was 38.1°C or higher, the intensity of this symptom is severe.

**Table 10:** Quarantine information.

C1	Were you in quarantine?	1. Yes 2. No
C2	If you answered yes in the previous question, where were you quarantined?	1. Home 2. Hospital 3. Hotel
C3	How long have you been quarantined?	1. Less than a week 2. A week 3. Two weeks 4. More than two weeks

## Data Availability

The data used to support the findings of this study are available from the corresponding author upon request.

## Appendix

Demographic information is shown in Table 8, post-recovery symptoms and symptoms duration are shown in Table 9, and quarantine information is shown in Table 10.
